# Application of Improved DEA Algorithm in Public Management Problem Classification

This article has been retracted.

**DOI:** 10.1155/2022/2568162

**Published:** 2022-09-19

**Authors:** Jialin Li

**Affiliations:** Vanderbilt University, Nashville, TN 37240, USA

## Abstract

In order to effectively solve the related problems in the process of public management, this research proposes an improved algorithm technology based on Data Envelopment Analysis (DEA) and classification algorithm. With the help of lever management, this paper further solves and overcomes the problem of DEA algorithm itself and the defect of “relative effectiveness.” At the same time, in order to avoid the impact on the input and output indicators, with the help of principal component analysis, taking the performance evaluation of public management departments as the research direction, this paper makes an empirical analysis on the performance evaluation of public management departments. The evaluation results of the index system show that the correlation coefficient between the efficiency value of the initial index system and the efficiency value of optimization 2 is 0.977759, and the correlation coefficient is less than 0.7. The evaluation results are more reasonable than those before the improvement.

## 1. Introduction

In recent years, with the continuous development of the market economy, the social governance structure has been continuously improved, and the pace of social governance has been gradually accelerated. As an important part of the process of social governance, the importance of public management is becoming more and more obvious. The so-called public management is the scientific management of public affairs, which includes the management of the government, administrative management, urban management, and other aspects. With the continuous deepening and development of public management in China, some major contradictions and problems begin to appear [1]. Such problems as insufficient practical operation means, insufficient governance ability, poor organizational personnel quality, and public management personnel training have seriously affected the improvement of the quality of public management [2–4]. This study is based on these issues, through the integration of Improved DEA algorithm to further improve the public management evaluation system.

On the basis of summarizing the above, foreign scholars elaborated the interaction between the transformation of government functions and the implementation of cultural policies. Xue put forward that only by adopting the overall governance mode, crossing over the administrative settings of each department, and realizing “horizontal” cross departmental cooperation can cultural services be truly implemented; otherwise, it will only be “a piece of empty talk” [5]; Zhao believes that the characteristic of cultural output is that with the growth of the national economy, the wage rate of the government's cultural department develops with other departments. However, due to the labor-intensive output, it is difficult for the productivity to keep pace with the wage growth rate, resulting in an increase in the cost of cultural input, which eventually leads to a doubling of public cultural expenditure [6]; Chen proposed that through the joint investment of the government and local cultural institutions, public cultural services can achieve twice the result with half the effort, and cause the domino effect, bringing more investment to cultural undertakings; joint investment requires both sides to express their own views and reach unity through consultation based on the principle of mutual cooperation and communication. Such a model is conducive to the diversity and innovation of public cultural development [7]; Ma European cultural identity, which involves ethnic and regional identity in a broader sense, is a model of self-understanding through which individuals, groups, and societies define themselves and their relationships with others. This changing relationship, in turn, will affect the change of self-understanding, that is, the difference in government system and environment will lead to the change of cultural identity [8].

In general, the lack of specialized research on the state of foreign service culture also means that research on the development of China's cultural service needs to be improved renewed in thought and action.

In China, DEA has been applied in many fields. National cotton mills, industryers, and smelters use the DEA method to evaluate the performance of companies and deliver the results to the actual department, which has been praised by stakeholders affected. The National Academic Association approached the DEA to evaluate its effectiveness, which was favored by many. The DEA is a great way to learn about the human resources and potential of coal production in China. Some scholars use the DEA method to determine that “finance is the most important factor affecting the performance of China's high-tech industry and human technology” [9]. He hoped that China's high-tech industry will continue to benefit from the application of science and technology of human resources in the field of performance measurement, innovation baking, and financial management. Some researchers have used the best data shell model to measure the performance of listed companies in the coal industry and estimate the market share and product shortages in the decision-making. They believe that the production efficiency of most listed coal enterprises is acceptable, but there are great individual differences. Many enterprises still have great room for improvement and put forward suggestions to the administrative departments [10].

## 2. Improved DEA Algorithm and Classification Algorithm

### 2.1. Improved DEA Algorithm and Its Application

There are designated decision-making units (DMUs) and design solutions (SU). Their sampling units and components have the same *M* input and output characteristics, and the input parameters and output parameters are as follows:

(1) $$\begin{array}{c} x_{p}={\left(x_{1p},x_{2p},\ldots ,x_{mp}\right)}^{T}\text{,} \end{array}$$

(2) $$\begin{array}{c} y_{p}={\left(y_{1p},y_{2p},\ldots ,y_{sp}\right)}^{T}\text{,} \end{array}$$

(3) $$\begin{array}{c} x_{j}={\left(x_{1j},x_{2j},\ldots ,{\bar{x}}_{mj}\right)}^{T}\text{,} \end{array}$$

(4) $$\begin{array}{c} y_{j}={\left(y_{1j},y_{2j},\ldots ,{\bar{y}}_{sj}\right)}^{T}\text{,} \end{array}$$

where equation (1) represents the value of the determination *p*, which includes the value of the measure; equation (2) represents the value of the p-order, resulting in the measured value; equation (3) represents the value of the *j*th cell at the input index value; equation (4) represents the value of the *j*th model unit of the output index value [11].

First, the production possibility set *T*(1) determined by the sample unit set is expressed as follows under the condition that the axiom system of the production possibility set of the sample unit and the decision-making unit is satisfied:

(5) $$\begin{array}{c} T\left(1\right)=\left\{\left.\left(x,y\right)\right|x\geq \overset{\bar{n}}{\underset{j=1}{\sum }}{\bar{x}}_{j}\lambda_{j},y\leq \overset{\bar{n}}{\underset{j=1}{\sum }}{\bar{y}}_{j}\lambda_{j},\delta \overset{\bar{n}}{\underset{j=1}{\sum }}\lambda_{j}=\delta ,\lambda =\left(\lambda_{1},\ldots ,\lambda_{\bar{n}}\right)\geq 0\right\}\text{,} \end{array}$$

where $\left({\bar{x}}_{j},{\bar{y}}_{j}\right)$ indicates the input and output status in the sample cell set. The input indicator reflects the consumed resources and is also the input data. The output indicator reflects the effectiveness and is the output data. According to the construction method of production frontier, the effective frontier of sample production possibility set *T*(1) is as follows:

**Assumption 1 .**

(6) $$\begin{array}{c} \bar{\omega },\bar{\mu },{\bar{\mu }}_{0}\;meet\;\bar{\omega }>0,\bar{\mu }>0\text{.} \end{array}$$

Hyperplane composed simultaneously:

(7) $$\begin{array}{c} L=\left\{\left.\left(x,y\right)\right|\omega^{-T}x-\mu^{-T}y-\delta {\bar{\mu }}_{0}=0\right\}\text{.} \end{array}$$

Meet the following set:

(8) $$\begin{array}{c} T\left(1\right)\subset \left\{\left.\left(x,y\right)\right|{\hat{\omega }}^{T}x-{\hat{\mu }}^{T}y-\delta {\hat{\mu }}_{0}\geq 0\right\},L\cap T\left(1\right)\neq \varphi \text{,} \end{array}$$

Then, the set represented by *L* is the effective surface of the sample possibility set *T*(1), and the intersection *L*∩*T*(1) is the effective frontier of the sample possibility set *T*(1).

There are now *n* decision-making units (DMUs) to be evaluated and *n* sample units selected. Both DMU and sample units have *m* input and *s* output indicators, which are expressed as follows:

(9) $$\begin{array}{c} x_{p}={\left(x_{1p},x_{2p},\ldots ,x_{mp}\right)}^{T}>0\text{,} \end{array}$$

(10) $$\begin{array}{c} y_{p}={\left(y_{1p},y_{2p},\ldots ,y_{sp}\right)}^{T}>0\text{,} \end{array}$$

(11) $$\begin{array}{c} x_{j}={\left(x_{1j},x_{2j},\ldots ,{\bar{x}}_{mj}\right)}^{T}>0\text{,} \end{array}$$

(12) $$\begin{array}{c} y_{j}={\left(y_{1j},y_{2j},\ldots ,{\bar{y}}_{sj}\right)}^{T}>0\text{,} \end{array}$$

Here, equation (9) represents the value of the input index and *p* is the unit value of the decision; formula (10) represents the output value and the unit value determined by *p*; formula (11) represents the value of the input index and the cell value of model *j*; formula (12) represents the output value and the *j*-type cell value [12].

The generalized CCR model for decision unit *p* is as follows:

(13) $$\begin{array}{c} \left(G-C^{2}R\right)\left\{\begin{array}{c} Maximize\;\mu^{T}y_{p}=V\left(d\right),\\ s.t\;\omega^{T}{\bar{x}}_{j}-\mu^{T}d{\bar{y}}_{j}\geq 0,j=1,\ldots ,\bar{m,}\\ \begin{array}{c} \omega^{T}x_{p}=1,\\ \mu ,\omega \geq 0,r=1,\ldots ,s;i=1,\ldots ,m, \end{array} \end{array}\right. \end{array}$$

where

(14) $$\begin{array}{c} \omega ={\left(\omega_{1},\omega_{2},\ldots ,\omega_{m}\right)}^{T}, \end{array}$$

(15) $$\begin{array}{c} \mu ={\left(\mu_{1},\mu_{2},\ldots ,\mu_{s}\right)}^{T}\text{.} \end{array}$$

Equation (14) represents the input index weight of the selected sample unit, equation (15) represents the output index weight of the selected sample unit, and *D* is a moving factor greater than 0.

The dual problem model of the generalized model can be expressed as follows:

(16) $$\begin{array}{c} \left(DG-C^{2}R\right)\left\{\begin{array}{c} \min\;\theta =D\left(d\right)\text{,}\\ s.t\overset{\bar{n}}{\underset{j=1}{\sum }}{\bar{x}}_{j}\lambda_{j}\leq \theta x_{p},\\ \overset{\bar{n}}{\underset{j=1}{\sum }}d{\bar{y}}_{j}\lambda_{j}\geq y_{p},\\ \lambda_{j}\geq 0,j=1,2,\ldots ,\bar{n.} \end{array}\right. \end{array}$$

The above formula can prove that (*G* − *C*^2^*R*) has an optimal solution.

### 2.2. Linear Separable Support Vector Classifier

Firstly, Lagrange function is introduced.

(17) $$\begin{array}{c} L\left(w,b,\alpha \right)=\frac{1}{2}{\left\|w\right\|}^{2}-\overset{l}{\underset{i=1}{\sum }}\alpha_{i}\left(y_{i}\left(\left(w\cdot x_{i}\right)+b\right)-1\right)\text{,} \end{array}$$

where

(18) $$\begin{array}{c} \alpha ={\left(\alpha_{1},\ldots ,\alpha_{l}\right)}^{T}\in R_{+}^{l}\text{.} \end{array}$$

The above formula is Lagrange multiplier. From the definition of duality, we can know that the minimum value of Lagrange function with respect to w, b must be obtained first. By extreme condition,

(19) $$\begin{array}{c} \Delta_{b}L\left(w,b,\alpha \right)=0,\Delta_{w}L\left(w,b,\alpha \right)=0\text{.} \end{array}$$

This leads to

(20) $$\begin{array}{c} \overset{l}{\underset{i=1}{\sum }}y_{i}\alpha_{i}=0\text{.} \end{array}$$

(21) $$\begin{array}{c} w=\overset{l}{\underset{i=1}{\sum }}y_{i}\alpha_{i}x_{i}\text{.} \end{array}$$

Bring equation (20) into equation (17) and use equation (21) to know that the dual problem of the original optimization problem can be expressed as

(22) $$\begin{array}{c} \max_{\alpha }-\frac{1}{2}\overset{l}{\underset{i=1}{\sum }}\overset{l}{\underset{j=1}{\sum }}y_{i}y_{j}\alpha_{i}\alpha_{j}\left(x_{i}\cdot x_{j}\right)+\overset{l}{\underset{j=1}{\sum }}\alpha_{j}\text{.} \end{array}$$

(23) $$\begin{array}{c} s.t\text{.}\overset{l}{\underset{i=1}{\sum }}y_{i}\alpha_{i}=0\;\alpha_{i}\geq 0,i=1,\ldots ,l\text{.} \end{array}$$

The algorithm we want can be obtained by converting the objective function into minimization.

## 3. Performance Evaluation of Public Management Cultural Service Classification Based on Improved DEA Algorithm

### 3.1. Construction of Index System

We check the impact of indicators on museum performance evaluation according to the commonality of specific indicators. The greater the degree of commonality, the greater the degree of common dependence of the index on the common factor, that is, it is relatively effective to use this common factor to explain the index. Correlation analysis is required before analysis [13]. Generally, the higher the correlation coefficient, the closer the relationship between the two index items. Generally speaking, above 0.7 can be understood as relatively high. By taking the data of 31 provinces in China from 2018 to 2021 as the sample data (124 sample data), after standardized processing, Spss21.0 was run to calculate the common factor, and the following results (Tables 1to 4) were obtained [14].

The analysis results of gravel diagram are shown in Figure 1.

Sample data passed KMO test. The higher the KMO value, the greater the significance of the changes and the greater the need for analysis. The chart shows that the KMO value is 0.879, indicating that the index is appropriate for analysis. In general, it is shown in Figure 1. Three indicators have been omitted due to differences in three indicators returned this year: cultural monuments, important artifacts, and the number of patents are less than 0.3. Go back to another measurement to get a performance measurement in time. Based on collaborations and releases, 10 museum performance measures were performed as shown in Table 5 [15].

It is scientific and innovative to use factor analysis to select the evaluation indicators of museums. Factor analysis is used to enhance the accuracy and objectivity of the index system [16]. In the actual operation of the museum, there are many and complex achievement indicators, but too many indicators are easy to form mutual interference between indicators, and it is difficult to find more accurate original data. Factor analysis method is used to eliminate some unnecessary and redundant indicators to achieve the purpose of simplification and optimization.

### 3.2. Performance Evaluation of Public Cultural Services Based on Methods

#### 3.2.1. Optimization of Input and Output Indexes Based on DEA Method

DEA method is based on known data sets, so the evaluation results directly depend on the selection of input and output indicators. In the chapter, the index system is constructed theoretically and scientifically, but the principle of the method itself on the data is not fully considered. Therefore, the index system should be analyzed from the perspective before performance evaluation. From the perspective of DEA application, the selection of DEA indicators should follow the following basic principles:

*Objective measurement*. When selecting a measuring device, whether the measurement objective can be achieved, i.e., the choice of the measuring device, the output measurement should be consistent with the functional and objective measurement. Objective assessment requires a variety of materials and tools to describe the whole process [17].

*Number of events*. Determine the number of units of measurement. Numerous input and output parameters can increase the number of positives, thereby reducing the effectiveness of the DEA method. Measurements should be kept as simple as possible at the target location. Some researchers believe that all input and output measures should not exceed 1/3 of the scoring sequence [18].

*Relevance*. Considering the relationship between input indicators and output indicators, the inputs and outputs of DMU are often not isolated [19]. When there is a strong linear correlation between an input indicator and other input indicators, it can be considered that the information of the indicator has been included by other indicators to a large extent, so it can be considered to exclude the input indicator. The same is true for output indicators. This will also lead to more DEA-effective units and affect the evaluation results.

*Diversity*. Since the core work of the method is “evaluation,” there are generally different aspects under a large evaluation objective. The diversity of input and output indicator systems should be considered [20]. Then, on the premise of determining the evaluation objective, multiple input and output indicator systems should be designed, such as from multiple indicators to fewer indicators, to observe which indicators have the greatest impact on the effectiveness value or design similar but different index systems to reflect different aspects of the evaluation.

The specific process is as follows: calculate the effective value of each decision-making unit through the practice index system and then calculate the effective value of each decision-making unit through the optimization index system that specifically reflects the evaluation purpose. Finally, the correlation coefficients of the two sets of effective values are calculated. If there is no significant correlation between the effective values calculated by the two index systems, it can be considered that the optimization index system is not comprehensive. On the contrary, if the correlation is significant, it indicates that the optimized index system can replace the previous index system for performance evaluation analysis [21]. The steps are as follows:

Step 1: determine the practice index system and preliminarily evaluate each decision-making unit; Step 2: optimize the index system based on principles and criteria and conduct preliminary evaluation on each decision-making unit; Step 3: calculate the correlation of the effectiveness values of the two sets of index systems obtained by the method and use the above criteria to judge the comprehensiveness and equivalence of the two sets of index systems so as to form a relatively accurate index system.

#### 3.2.2. Principle of Determining Index Weight

*(1) The principle of system optimization*. In the evaluation index system, each index has its role and contribution to the system and has its importance to the system. Therefore, the determination of index weight should not only start from a certain index but should consider comprehensively, deal with the relationship between the evaluation indexes, and reasonably allocate their weights. We should follow the principle of system optimization and take the overall optimization as the starting point and goal. Under the guidance of this principle, analyze and compare each evaluation index in the evaluation index system, weigh their respective roles and effects on the whole, and then judge their relative importance. Determine their respective weights, that is, they cannot be evenly distributed, nor can they unilaterally emphasize the optimization of a certain index or a single index while ignoring the development of other aspects. In practice, each indicator should play its due role.

*(2) The principle of combining the subjective intention of the evaluator with the objective situation*. The weight of the evaluation index reflects the guiding intention and values of the evaluator and the organization. When they feel that a certain indicator is very important and need to highlight its role, they must use a larger weight for each indicator. However, the actual situation is often not completely consistent with people's subjective will. For example, when determining the weight, we should consider the following issues: historical indicators and realistic indicators, recognized by the society and the particularity of the enterprise, and balance between the same industry and the same type of work. Therefore, we must consider the reality at the same time and combine the guiding intention with the reality. As mentioned earlier, economic and social benefits should be considered simultaneously in evaluating the performance of public cultural services.

*(3) The principle of combining democracy with centralism*. Weight is people's understanding of the importance of evaluation indicators, is the quantification of qualitative judgment, and is often affected by personal subjective factors. Different people have their own views on the same thing, and they are often different, in which there are reasonable elements. Of course, there are also prejudices caused by personal values, abilities, and attitudes. This requires the implementation of the principle of group decision-making, integrating the opinions of relevant personnel to complement each other and form a unified plan. This process has the following advantages: considering problems comprehensively, making the weight distribution more reasonable, and preventing individuals from understanding and dealing with problems unilaterally. It objectively coordinates the contradictions of different opinions among the evaluation parties. The scheme determined through discussion, consultation, and investigation of various specific situations is very persuasive and eliminates many unnecessary disputes in advance. This is a mode of participating in management. During the discussion of the scheme, all parties put forward their own opinions and have further experience and understanding of the evaluation objectives and system objectives. In daily work, they can better work according to the original objectives [22].

The standard values of qualitative indicators are different from those of quantitative indicators, which are easy to collect. They are generally obtained through the following methods:

*(1) Expert experience*. Expert experience refers to the experience of experts in judging the performance of the public resource supply based on their own experience, combining the political and economic development situation at that time, as well as the economic and social benefits generated by similar projects, units, or departments using similar funds in previous years, and combining certain domestic and foreign experience.

The questionnaire test establishes qualitative standards through public judgment for some indicators related to public satisfaction and expenditure targets to be achieved.

*(2) Horizontal comparison*. Make a comprehensive comparison of the results achieved by the supply performance of similar public goods at home and abroad. Of course, with the continuous progress of science and technology in human society, new technologies and methods will continue to emerge, and some qualitative indicators that are difficult to quantify will be gradually quantified or accurately grasped.

#### 3.2.3. Performance Evaluation Method System of Public Cultural Services

When engaging in any work, we must understand the methods. As the resource input of public cultural services depends on the government and financial input, the output mainly depends on the public's awareness and satisfaction with culture. As a result, the competition mechanism in the whole field is not strong, and public cultural services are difficult to quantify. In particular, the public cultural services studied in this paper are difficult to measure by market means. In addition, the authenticity and comparability of data in the field of cultural public services and the difficulty in quantifying most of the achievements of cultural services make it difficult to measure the performance of the public sector. Despite this, people still try to apply various advanced methods to the performance evaluation of public cultural services. The main methods are as follows:

*(1) Performance evaluation table method*. The performance evaluation table method, also known as the scoring table method, should be said to be an early method. It mainly uses the relevant performance factors formulated by the government to evaluate the performance of the work (such as the number of annual visitors to the museum and the number of books lent out). Compare and score the work performance with the relevant factors one by one and then get the overall results of the work performance. According to the results, it is classified into four levels: excellent, good, qualified, and unqualified.

*(2) Management by objectives*. It is the most typical result-oriented performance evaluation method. At that time, the objective management method was widely used. The evaluation object of the objective management method was mainly the work performance of employees, that is, focusing on the completion of objectives. Through this method, employees could be promoted to work towards objectives to a certain extent.

*(3) Key performance indicator method*. The theoretical basis of the process of measuring performance is based on the “February 8 principle” stated by Italian scientist Pareto. In the process of establishing the business value, it is believed that 80% of the work of each department and staff do 20% of the simple behavior, and this 20% capture will understand all. Along with these concepts, key indicators such as feedback and benefits of the organization's internal processes are identified, modeled, accounted for, evaluated, and implemented, and goals of the industry have exploded. This way, it is possible to clearly identify the key roles of responsibility to the director of the company and to develop standards of performance for the employees in the department.

*(4) Data envelopment analysis method*. Data envelopment analysis (DEA) is developed on the basis of the theory of “relative efficiency evaluation.” Its core idea is to estimate the frontier of effective production by observing a group of values about input and output. It is applicable to the effectiveness evaluation of multiple decision-making units with the same type of multiple inputs and outputs. DEA has obvious advantages in efficiency evaluation: first, in the process of evaluation, only input indicators and output indicators need to be determined, without constructing specific production functions or models; secondly, it is suitable for complex objective evaluation with multiple inputs and outputs; then, this method does not require the dimension of the indicators. As long as a specific indicator of the decision-making unit uses the same dimension, the original data can be directly analyzed. The above advantages of DEA method can just meet the requirements of efficiency evaluation of public cultural services. First of all, the government's human, financial, and material inputs in various branches of public cultural services are eventually transformed into various specific public goods and services. Generally, we can only determine which outputs are related to inputs. As for the transformation relationship behind it, it is difficult to quantify and measure in reality; secondly, public cultural services cover a wide range, which belongs to a typical multi-input and multi-output situation.; Moreover, it is inconvenient or impossible to measure the input and output of public cultural service supply in terms of money or some other specific dimension in many cases, and DEA can just avoid this point. Therefore, the DEA method will have a broad application prospect in evaluating the efficiency of government supply of public goods. This paper is also based on this discussion.

#### 3.2.4. Classification Performance Evaluation of Public Cultural Services Based on *C*^2^*R* Model

First of all, according to the important position of museums, public libraries, and mass art centers in public cultural services, the practice index system has been established according to the fifth chapter. Then, according to the optimization idea of input and output indicators based on DEA method, the practice indicator system is optimized to form a new indicator system, and the performance structure model diagram of public cultural services is constructed as shown in Figure 2.

Finally, two sets of index systems are input through model *C*^2^*R* for operation to form the corresponding performance evaluation result analysis. The flow chart of public cultural service classification performance evaluation based on *C*^2^*R* model is shown in Figure 3.

## 4. Performance Evaluation of Public Cultural Service Classification Based on *C*^2^*R* Model

### 4.1. Determination of Input and Output Indicators

The indicator system constructed according to the above is shown in Table 6.

According to the optimization of input and output indicators of the above DEA method, since the employees' indicators already include the indicators of senior employees, the senior employees are eliminated from the perspective of simplification. Similarly, the actual use of the housing area index already includes the exhibition room index, so the exhibition room is excluded. In the output indicators, the number of visits by minors has been reflected in the number of visitors, so the number of minor visits is excluded. The index system after comprehensive optimization is shown in Table 7.

*C* ^2^ *R* model is used to calculate the data of the two groups of index systems, and the efficiency value is obtained as shown in Table 8.

It cannot be found from the table that the optimized index system has a great impact on some regions, in which the effective value of Beijing is reduced from relatively effective 1 to 0.48, which indicates that the index items subject to subdivision have a great impact on the performance value [23]. The correlation coefficient obtained from the correlation test of the effective values corresponding to the two groups of index systems is 0.644816. We believe that if the correlation coefficient is greater than 0.7, then our optimized index system cannot replace the original index system. Therefore, it is necessary to further optimize the practice performance evaluation indicators, find out which indicator system has a greater impact, and conduct correlation analysis on the original indicator system as shown in Table 9.

The removed senior staff and exhibition rooms are highly correlated, and the correlation value between the number of collections and other indicators is mostly below 0.7. Therefore, the optimization indicators are re-optimized as shown in Table 10.

*C* ^2^ *R* model is used to calculate the data of the two groups of indicator systems, and the effective values obtained are shown in Table 11. The correlation coefficient obtained from the correlation test of the effective values corresponding to the two groups of index systems is 0.903433. We believe that if the correlation coefficient is greater than 0.7, then our secondary optimized index system cannot replace the original index system. Through the optimization of indicators, the indicators after the secondary optimization of museum performance evaluation can relatively comprehensively represent the indicators of museum performance evaluation. The following analysis is also based on the indicators after the secondary optimization.

### 4.2. Performance Evaluation Analysis

In the previous section, the efficiency values of provinces are calculated according to the evaluation secondary optimization indicators. After processing, see Figure 4.

The overall service efficiency of national museums will be moderate in 2020. The efficiency level of the national evaluation is 0.870559, and the overall efficiency is moderate. This has something to do with the country's great investment in public cultural undertakings in recent years. However, there are some regions with low efficiency and relatively poor efficiency in Xinjiang and Ningxia. The projection analysis is shown in Table 12, and the investment needs to be adjusted. Through the above index adjustment, we can also find that the number of collections is a very important index item for museums. In the future construction and development of museums, museums should devote more energy to how to enrich the number of collections in museums.

The regional characteristics of museum performance evaluation are obvious. Among the 31 provinces, autonomous regions, and municipalities directly under the central government in the mainland of China, 14 regions' museum performance is efficient compared with other regions, including Beijing, Tianjin, Shanghai, Hubei, and Anhui. Liaoning, Ningxia Hui autonomous region, Shaanxi, and Gansu have relatively low-efficiency values. The results show obvious regional characteristics.

The low number of collections is the main reason for the low efficiency in some areas, which has been fully reflected in the process of index optimization. Therefore, to improve the efficiency of museums, on the one hand, it is necessary to increase the number of collections, exhibitions, and other measures, on the other hand, it is necessary to make reasonable allocation in terms of employees, financial allocation, and the actual use of housing area.

## 5. Conclusion

Based on the improved DEA algorithm, this research puts forward the theoretical framework of public cultural service performance evaluation system. The theoretical framework of performance evaluation system is the key to the government supply of public cultural services. The construction of the public cultural service performance evaluation index system needs to have a clear target, be good at using scientific analysis methods, scientifically measure the validity and reliability of the index system, and design the public cultural service performance evaluation index system according to the objectives, performance dimensions, performance orientation, and other ideas of performance evaluation. *C*^2^*R* model and superefficiency model in DEA algorithm are innovatively and comprehensively applied to the performance evaluation of government supply of public cultural services. DEA method has many advantages. It determines the attribution of the index system by fitting the path coefficients of each factor in the model through objective data and automatically generates weights. It is suitable for analyzing the performance evaluation of public cultural services. On the basis of collecting a large number of statistical sample data, taking into account the large differences between different types of public cultural services, this paper makes an empirical analysis on the performance appraisal of public management departments with the help of principal component analysis and taking the performance appraisal of public management departments as the research direction. The evaluation results of the index system show that the correlation coefficient between the efficiency value of the initial index system and the efficiency value of optimization 2 is 0.977759, and the correlation coefficient is less than 0.7. The evaluation results are more reasonable than those before the improvement. It can be seen that this method improves the rationality and reliability. The general performance evaluation is used to regard the categories of the total performance that are actually intrinsically related as uncorrelated individuals for analysis. Therefore, this paper uses the superefficiency model to evaluate the overall performance of public cultural services and gives the interaction between the input and output indicators of public cultural services. The basic conclusion of the government supply performance of public cultural services in China is that the overall performance is insufficient, the regional gap is large, the structure is balanced, and the economic support is obvious.

## Figures and Tables

**Figure 1:** Gravel diagram.

**Figure 2:** Performance structure model of public cultural services.

**Figure 3:** Flow chart of public cultural service classification performance evaluation.

**Figure 4:** Line chart of museum performance evaluation.

**Table 1:** Sample statistics.

	Mean value	Standard deviation	Analysis N
Employees/person	1948.099	1427.7271	124
Senior title	115.639	81.6104	124
Financial appropriation/thousand yuan	250456.422	196399.2388	124
Collection pieces/set	527715.645	397193.3103	124
Number of cultural relics restored this year/set	1088.343	2128.6877	124
Basic display	295.776	571.9660	124
Hold exhibitions	329.343	274.4959	124
Minor visitors/1000	3912.25414523495100	3214.33641453795100	124
Number of visitors/1000	13687.29044512312100	11149.19042516372100	124
Patent	2.487	6.2203	124
Number of completed projects	6.451	8.3224	124
Exhibition room/1000 square meters	173.34782384712390	139.74732354212390	124
Actual floor area/10000 square meters	365.44756383712250	268.74345533717250	124

**Table 2:** KMO and Barrett tests.

Kaiser–Meyer-01kin measure of sampling adequacy		.876
Bartlett's sphericity test	Approximate chi-square	1672.043
	df	78
	Sig.	0.000

**Table 3:** Common factor variance 1 principal component analysis.

	Initial	Extract
Employees/person	1.000	0.654
Senior title	1.000	0.691
Financial appropriation/thousand yuan	1.000	0.666
Collection pieces/set	1.000	0.653
Number of cultural relics restored this year/set	1.000	0.193
Basic display	1.000	0.077
Hold exhibitions	1.000	0.757
Minor visitors/1000	1.000	0.732
Number of visitors/1000	1.000	0.894
Patent	1.000	0.234
Number of completed projects	1.000	0.631
Exhibition room/1000 square meters	1.000	0.821
Actual floor area/10000 square meters	1.000	0.921

**Table 4:** Common factor variance principal component analysis.

Ingredients	Initial eigenvalue			Extract sum of squares load		
	Total	Variance%	Cumulative%	Total	Variance%	Cumulative%
1	7.943	61.161	61.161	7.943	61.161	61.161
2	0.993	7.612	68.774			
3	0.978	7.531	76.213			
4	0.743	5.682	81.943			
5	0.621	4.634	86.876			
6	0.454	3.421	90.122			
7	0.412	3.139	93.201			
8	0.271	2.008	95.212			
9	0.258	1.921	97.136			
10	0.191	1.446	98.599			
11	0.131	.994	99.601			
12	0.034	.241	99.846			
13	0.023	.167	100.00			

**Table 5:** Practical indicators of museum performance evaluation.

Indicator classification	Indicator name
Input indicators	Employees
	Senior title
	Financial appropriation
	Number of collections
	Actual floor area

Output indicators	Number of collections
	Hold exhibitions
	Number of visitors
	Number of completed projects
	Minor visitors

**Table 6:** Museum performance evaluation index system.

Indicator classification	Indicator name
Input indicators	Employees
	Senior title
	Financial appropriation
	Exhibition room
	Actual floor area

Output indicators	Number of collections
	Hold exhibitions
	Number of visitors
	Number of completed projects
	Minor visitors

**Table 7:** Optimization indicators for museum performance evaluation.

Indicator classification	Indicator name
Input indicators	Employees
	Financial appropriation
	Actual floor area

Output indicators	Hold exhibitions
	Number of visitors
	Number of completed projects

**Table 8:** Cross-value comparison of two index systems.

NO.	DMU	Score	Score-optimize1
1	Beijing	1	0.480356868
2	Tianjin	1	0.537980302
3	Hebei province	0.839556	0.758941004
4	Shanxi province	0.810403	0.552091004
5	Inner Mongolia autonomous region	0.669882	0.568362204
6	Liaoning province	0.486929	0.423907129
7	Jilin province	1	1
8	Heilongjiang province	1	1
9	Shanghai	1	0.532312132
10	Jiangsu province	1	0.973383461
11	Zhejiang province	0.828156	0.799626211
12	Anhui province	1	1
13	Fujian province	0.98733	0.985527088
14	Jiangxi province	0.76535	0.697399767
15	Shandong province	0.908386	0.881542336
16	Henan province	0.921388	0.921406465
17	Hubei province	1	0.834135771
18	Hunan province	1	1
19	Guangdong province	0.92253	0.898512197
20	Guangxi Zhuang autonomous region	0.734522	0.670123232
21	Hainan	1	1
22	Chongqing city	0.966883	0.895422931
23	Sichuan province	1	0.889086523
24	Guizhou province	1	1
25	Yunnan province	1	1
26	Tibet autonomous region	1	1
27	Shaanxi province	0.65188	0.485806762
28	Gansu province	1	0.592953371
29	Qinghai province	1	0.987601029
30	Ningxia Hui autonomous region	0.568312	0.561783341
31	Xinjiang Uygur autonomous region	0.795216	0.703376021

**Table 9:** Correlation analysis of museum index system.

	Employees (person)	Senior title	Financial appropriation (thousand yuan)	Exhibition room (thousand square meters)	Actual floor area (ten thousand square meters)	Number of collections (piece/set)	Hold exhibitions	Number of visitors (thousand)	Number of completed projects	Minor visitors (1000)
Employees (person)	1.00	0.80	0.77	0.87	0.91	0.67	0.76	0.91	0.73	0.78
Senior title	0.81	1.00	0.71	0.84	0.87	0.72	0.82	0.77	0.65	0.66
Financial appropriation (thousand yuan)	0.79	0.72	1.00	0.71	0.81	0.78	0.65	0.67	0.71	0.51
Exhibition room (thousand square meters)	0.85	0.83	0.67	1.00	0.96	0.67	0.92	0.93	0.67	0.84
Actual floor area (ten thousand square meters)	0.90	0.87	0.80	0.98	1.00	0.75	0.92	0.95	0.73	0.82
Number of collections (piece/set)	0.67	0.71	0.78	0.65	0.74	1.00	0.58	0.63	0.61	0.51
Hold exhibitions	0.77	0.82	0.65	0.89	0.89	0.61	1.00	0.87	0.73	0.81
Number of visitors (1000)	0.88	0.77	0.71	0.91	0.92	0.64	0.87	1.00	0.73	0.91
Number of completed projects	0.71	0.67	0.72	0.67	0.77	0.64	0.73	0.74	1.00	0.56
Minor visitors (1000)	0.78	0.63	0.51	0.83	0.81	0.49	0.81	0.94	0.54	1.00

**Table 10:** Secondary optimization indicators for museum performance evaluation.

Indicator classification	Indicator name
Input indicators	Employees
	Financial appropriation
	Actual floor area

Output indicators	Hold exhibitions
	Number of visitors
	Number of completed projects
	Number of collections

**Table 11:** Efficiency values of two indicator systems.

NO.	DMU	Score	Score-optimization1
1	Beijing	1	1
2	Tianjin	1	1
3	Hebei province	0.839556	0.758941004
4	Shanxi province	0.810403	0.702091004
5	Inner Mongolia autonomous region	0.669882	0.668362204
6	Liaoning province	0.486929	0.483907129
7	Jilin province	1	1
8	Heilongjiang province	1	1
9	Shanghai	1	1
10	Jiangsu province	1	1
11	Zhejiang province	0.828156	0.829626211
12	Anhui province	1	1
13	Fujian province	0.98733	0.985527088
14	Jiangxi province	0.76535	0.697399767
15	Shandong province	0.908386	0.901542336
16	Henan province	0.921388	0.921406465
17	Hubei province	1	1
18	Hunan province	1	1
19	Guangdong province	0.92253	0.898512197
20	Guangxi Zhuang autonomous region	0.734522	0.730123232
21	Hainan	1	1
22	Chongqing city	0.966883	0.955422931
23	Sichuan province	1	0.909086523
24	Guizhou province	1	1
25	Yunnan province	1	1
26	Tibet autonomous region	1	1
27	Shaanxi province	0.65188	0.602806762
28	Gansu province	1	0.641953371
29	Qinghai province	1	1
30	Ningxia Hui autonomous region	0.568312	0.561783341
31	Xinjiang Uygur autonomous region	0.795516	0.703376061

**Table 12:** Projection analysis of museum performance evaluation.

30	Ningxia Hui autonomous region	0.5617833			
	Employees (person)	208	117.41343	−91.587372	−43.81%
	Financial appropriation (thousand yuan)	50246	28227.801	−22019.123	−43.81%
	Housing area (10000 square meters)	66.17	36.417263	−29.761824	−44.98%
	Hold exhibitions	43	43	0	0.00%
	Number of visitors (thousand)	840.10	840.10	0	0.00%
	Completed projects	0	0.6316811	0.6316811	999.90%

31	Xinjiang Uygur autonomous region	0.7023741			
	Employees (person)	853	599.27271	−252.73361	−29.61%
	Financial appropriation (thousand yuan)	126345	88875.084	−37479.921	−29.61%
	Housing area (10000 square meters)	205.61	117.38304	−87.237841	−42.64%
	Hold exhibitions	183	182	0	0.00%
	Number of visitors (thousand)	6073.74	6073.74	0	0.00%
	Completed projects	1	6.6904798	5.6905199	569.05%

## Data Availability

The data set can be obtained from the author upon request.
